# Identification of Protein Expression Changes in Hepatocellular Carcinoma through iTRAQ

**DOI:** 10.1155/2020/2632716

**Published:** 2020-01-23

**Authors:** Yuanyuan Zhang, Xia Ying, Qian Zhao, Jinlu Ma, Dan Zhang, Chenchen He, Suxia Han

**Affiliations:** ^1^Department of Pediatrics, The First Affiliated Hospital, Xi'an Jiaotong University, Xi'an 710061, China; ^2^Department of Gynecology and Obstetrics, Women's Hospital, Zhejiang University School of Medicine, Hangzhou 310006, China; ^3^Department of Ear Nose Throat Pharynx, The First Affiliated Hospital, Xi'an Jiaotong University, Xi'an 710061, China; ^4^Department of Oncology, The First Affiliated Hospital, Xi'an Jiaotong University, Xi'an, Shaanxi 710061, China; ^5^Department of Cell Biology and Genetics, School of Basic Medical Sciences, Xi'an Jiaotong University Health Science Center, Xi'an 710061, China

## Abstract

**Background:**

Hepatocellular carcinoma (HCC) is a malignant tumor associated with a poor prognosis. Serum biomarkers of HCC have the potential to improve the diagnosis, provide a means to monitor the tumors, and predict their malignancy. Proteins that are expressed differentially between HCC patients and normal controls have the potential to be biomarkers.

**Method:**

Serum samples from 10 confirmed HCC patients and 10 controls were collected. The differentially expressed proteins in the serum were identified using an isobaric tags for relative and absolute quantitation- (iTRAQ-) based method. Potential serum biomarkers were validated by ELISA in another 20 HCC patients and 20 controls. Their expression data in HCC were extracted from The Cancer Genome Atlas (TCGA) dataset.

**Results:**

A total of 260 proteins were measured in the serum of HCC patients and compared to those in sex- and age-matched normal controls. Forty-one proteins displayed significant changes, with 26 being downregulated and 15 being upregulated. Upregulated proteins included alpha-1-antitrypsin (A1AT) and peroxiredoxin 2 (PRDX2), and downregulated proteins included paraoxonase 1 (PON1) and C-reactive protein (CRP). We then used ELISA to measure serum levels of A1AT, PRDX2, PON1, and CRP in another 20 patients with HCC and found that only PON1 levels were consistent with the iTRAQ result. In TCGA dataset, PON1 expression was downregulated in HCC tissues (*P* < 0.001) and low expression of PON1 was associated with poor survival in HCC patients (*P* < 0.001) and low expression of PON1 was associated with poor survival in HCC patients (

**Conclusions:**

PON1 could act as a biomarker for HCC to assist in the diagnosis of HCC.

## 1. Introduction

Hepatocellular carcinoma (HCC) is an invasive tumor associated with high incidence and mortality. Serum biomarkers are considered to be of potential value in the diagnosis and monitoring of various diseases, including tumors, because their measurement is convenient and minimally invasive. The vast majority of HCC is diagnosed at advanced stages, resulting in high mortality rates that could be reduced through early detection using serum biomarkers.

Proteomics is the study and characterization of proteins on a large scale. It is a powerful way for biomarker discovery. Several promising biomarkers for HCC have been identified using proteomic approaches. Using the isobaric tags for relative and absolute quantitation- (iTRAQ-) based quantitative proteomics, Xing et al. showed that HSD17B13 and HK2 might be promising biomarkers for the primary HCC with single and multiple lesions [1]. And He et al. identified 14 proteins as potential serum biomarkers for AFP-negative HBV-related HCC [2]. In this study, we detected proteins that are differentially expressed in HCC patient serum samples using an iTRAQ-based method. In total, 41 differentially expressed proteins were identified. We selected 4 proteins for further verification and found that only paraoxonase 1 (PON1) might be a potential serum biomarker for HCC. However, additional studies that recruited more patient samples were required to validate the results for differentially expressed proteins reported in this manuscript.

## 2. Materials and Methods

### 2.1. Patient Samples

Blood from 10 HCC patients and 10 healthy controls for iTRAQ was sampled after obtaining informed consent and approval from the First Affiliated Hospital of Xi'an Jiaotong University. And then, serum from another 20 HCC patients and 20 healthy controls for ELISA was collected from the First Affiliated Hospital of Xi'an Jiaotong University. The demographic data, etiologies, comorbidities, and HCC characteristics are summarized in Table 1. There was no significant difference in gender and age distribution between the two groups. All patients in this study underwent curative surgery for the removal of tumors that were histologically confirmed as HCC. They had not undergone radio- or chemotherapy before. Control serum samples were obtained from age- and sex-matched individuals with no prior health conditions. Serum samples were separated and stored immediately at -80°C.

### 2.2. Sample Preparation, iTRAQ Labeling, and Mass Spectrometry

Serum pools were depleted of most abundant proteins using an Agilent Human 14 Multiple Affinity Removal System Column following the manufacturer's instruction. Ultrafiltration tubes (10 kDa, Sartorius) were used for desalination and concentration of low-abundance components. Protein in the supernatant was assayed with a BCA Protein Assay Kit (Bio-Rad, USA). The protein (20 *μ*g) from each sample was mixed with 5X loading buffer and separated on a 12.5% SDS-PAGE gel and visualized by Coomassie Blue R-250 staining. A filter-aided sample preparation (FASP) [3] was used to remove the detergent, DTT, and other low molecular weight components and digest the proteins. One hundred micrograms of each peptide mixture was labeled using an iTRAQ reagent 8-plex kit (SCIEX, Framingham, MA) according to the manufacturer's instructions. iTRAQ-labeled peptides were fractionated by Strong Cation Exchange (SCX) chromatography using the AKTA purifier system (GE Healthcare). Each fraction was injected for nano-LC-MS/MS analysis. High-resolution LC-MS/MS analysis was performed on a Q Exactive mass spectrometer (Thermo Fisher Scientific) operated in a positive ion mode that was coupled to an EASY-nLC liquid chromatograph (Thermo Fisher Scientific). The MS data were acquired in a data-dependent acquisition mode. The top 20 precursor ions were selected from each MS full scan in the HCD collision cell. The instrument was run with the peptide recognition mode enabled. The raw files were processed using Proteome Discoverer 1.4 (Thermo Scientific) and searched using the Mascot search engine (version 2.2, Matrix Science) against the UniProt protein human database (134,919 sequences). The false discovery rate (FDR) for peptides was set to 1%.

### 2.3. Enzyme-Linked Immunosorbent Assay (ELISA)

The human A1AT ELISA kit (KE00037, Proteintech Group, Wuhan, China), human PRDX2 ELISA kit (DY3489-05, R&D System, Minneapolis, USA), human PON1 ELISA kit (DYC5816-2, R&D System, Minneapolis, USA), and human CRP ELISA kit (KE00004, Proteintech Group, Wuhan, China) were used for the detection of the levels of alpha-1-antitrypsin (A1AT), peroxiredoxin 2 (PRDX2), paraoxonase 1 (PON1), and C-reactive protein (CRP) according to the manufacturer's instructions.

### 2.4. Statistical Analysis

Continuous data was tested for normality by the Kolmogorov-Smirnov test. Normal distribution variables are presented as the mean ± standard deviation (SD) and compared by the Student *t*-test. Abnormal distribution variables are presented as medians (interquartile range (IQR)) and compared by the Mann-Whitney rank-sum test. Categorical variables were presented as absolute numbers and/or percent frequencies and compared by the chi-square test or Fisher's exact test, as appropriate. All of the statistical analyses were performed with SPSS software (version 18.0; SPSS Inc., Chicago, IL, United States). A two-tailed *P* value < 0.05 was considered statistically significant.

### 2.5. TCGA Data Extraction

A1AT, PRDX2, PON1, and CRP expression and clinicopathological parameters in HCC patients were downloaded from The Cancer Genome Atlas (TCGA, https://tcga-data.nci.nih.gov/tcga) data portal. The expression level of each gene was compared between HCC tissues and noncancer tissues. Based on the FPKM value of each gene, patients were classified into two expression groups and the correlation between the expression level and patient survival was examined. The prognosis of each group of patients was examined by Kaplan-Meier survival estimators, and the survival outcomes of the two groups were compared by log-rank tests. Maximally separated Kaplan-Meier plots are presented. A log rank *P* value < 0.001 in maximally separated Kaplan-Meier analysis was considered statistically significant.

## 3. Results

### 3.1. Differential Expression Analysis of Serum Proteins between HCC and Healthy Controls Using iTRAQ

As shown in Figure 1(a), a total of 260 proteins were detected from the samples. Using the cutoff threshold of >1.2 or <0.8 and 95% confidence at a 1% FDR [4], we identified 41 proteins which displayed significantly different expression levels between HCC patients and healthy controls. Among them, 26 were downregulated and 15 were upregulated (Table 2).

### 3.2. GO Annotation and Functional Classification for Differentially Expressed Proteins

The Gene Ontology (GO) enrichment analysis showed that these differentially expressed proteins were mostly located in the cytoplasm, extracellular matrix, organelle, and macromolecular complex (Figure 1(b)). They were associated with 296 different molecular functions (Figure 1(c)). Most were involved in responses to stimuli and regulation of biological, metabolic, or developmental processes. Based on a cluster of orthologous groups of proteins (COG), these differentially expressed proteins could be classified into seven functional groups including binding activity, catalytic activity, transporter activity, and enzyme regulation (Figure 1(d)).

### 3.3. KEGG Automatic Annotation Server Analysis of Pathways for Differentially Expressed Proteins

Because biochemical reactions are achieved by different cooperative protein interactions, a KEGG pathway analysis was performed. In our study, differentially expressed proteins with significant matches were assigned to known KEGG metabolic or signaling pathways.  Figure 1(e) shows the KEGG pathways involved by the differentially expressed proteins. The most abundant ones included complement and coagulation cascades (7 members) and the Staphylococcus aureus infection pathway (4 members).

### 3.4. Validation of Differentially Expressed Proteins in HCC Serum Using ELISA

To validate the iTRAQ results, ELISA was used to measure four candidate proteins, A1AT, PRDX2, PON1, and CRP, in the serum of another 20 HCC patients and 20 healthy controls. As shown in Figures 2(a)–2(d), A1AT and PON1 levels were significantly decreased and CRP levels were significantly increased in HCC patients. There was no significant difference in serum PRDX2 levels between HCC patients and healthy controls. Thus, only PON1 levels were consistent with the iTRAQ result (Table 1).

### 3.5. A1AT, PRDX2, PON1, and CRP Expression in HCC in TCGA Database

A total of 374 HCC cases and 50 non-HCC cases were included in TCGA data. As shown in Figures 3(a)–3(d), A1AT, PON1, and CRP were downregulated and PRDX2 was upregulated in HCC tissues compared with noncancer tissues (*P* < 0.001). To evaluate the prognostic value of A1AT, PRDX2, PON1, and CRP in HCC, the expression levels were divided into the high-expression group and the low-expression group. The maximally separated Kaplan-Meier plots are presented in Figures 4(a)–4(d). Only PON1 expression was a significant prognostic factor for the overall survival in TCGA cohort. Low expression of PON1 was associated with poor survival in HCC patients (*P* < 0.001).

## 4. Discussion

We investigated the serum proteome profiles of HCC patients compared to normal controls in an attempt to develop a noninvasive diagnostic test for HCC. In addition, we conducted an in-depth study on hepatic proteins. Using an iTRAQ-based two-dimensional LC-MS/MS serum profiling method, we identified 41 differentially expressed proteins in HCC patients. These proteins were associated with protease inhibition, protein-secretion regulation, antioxidation, tumor control, and lipid metabolism.

Among the 41 differentially expressed proteins, we selected A1AT, PRDX2, PON1, and CRP for further verification. We selected these 4 proteins because they have not been confirmed as HCC biomarkers and their functions are closely related to liver diseases.

A1AT is a 52 kDa protein and a member of the serpin family. It is the most abundant liver-derived glycoprotein in the plasma [5]. The main function of A1AT is to inhibit neutrophil elastase and other serine proteases, including proteinase-3 and plasmin activator [6]. Elevated levels of A1AT have been proposed to discriminate cancer from chronic benign diseases and clinical remission from relapse [7]. A recent proteomic study showed marked divergence in A1AT expression between HCC tissue samples and precancerous lesions, suggesting that alterations in A1AT expression occur frequently during the development of HCC [8]. Serum A1AT levels in patients with HCC were significantly higher than those in patients with liver cirrhosis or chronic hepatitis [9]. The production of A1AT by tumor cells correlates with regional proteolytic and inflammatory activity that may be involved in the protection of tumor cells [10]. Elevated A1AT levels were proposed as a diagnostic and prognostic marker of HCC [11]. However, A1AT gene expression was significantly downregulated in TCGA database. In our current study, serum A1AT was significantly increased as measured by iTRAQ, but decreased as measured by ELISA. The discrepancy may be related to the small sample size in our study. However, it is also possible that A1AT might not be a good biomarker for HCC.

PRDX2 is an antioxidant enzyme which reduces hydrogen peroxide and alkyl hydroperoxides. It is a chemotherapy responsiveness biomarker for osteosarcoma [12]. PRDX2 inhibits TNF-*α*-induced apoptosis in HCC cells and reduces ROS generation and cell death during oxidative stress [13]. In screening for new plasma biomarkers for liver disease, Lu et al. found that PRDX2 is a potential biomarker for early diagnosis of HBV-related liver fibrosis [14]. In TCGA dataset, PRDX2 gene expression was upregulated in HCC tissues. However, PRDX2 is not a good prognostic marker for HCC. In the iTRAQ analysis, we found that PRDX2 levels were increased in HCC patients. But this result could not be confirmed by ELISA in another set of HCC samples. Thus, whether PRDX2 is not a good candidate for serum biomarkers of HCC warrants further investigation.

PON1, a high-density lipoprotein- (HDL-) associated protein, is known to contribute to cancer development [15]. PON1 was found to be a potential marker of survival in patients with breast cancer recurrence [16]. It is a liver-induced glycoprotein enzyme responsible for protection against reactive oxygen species and inflammation and has been associated with various cancers. PON1 may also be a risk factor for chronic hepatitis B [17], and glycan differences in serum PON1 may serve as potential biomarkers to distinguish early HCC from liver cirrhosis [18]. In this study, we have shown that PON1 expression was significantly decreased in HCC using iTRAQ-based serum proteomic analysis. This result was confirmed by ELISA in another set of HCC samples. Analyzing the data in TCGA database also showed that PON1 gene expression was downregulated in HCC tissues and low expression of PON1 was associated with poor survival in HCC patients. Taken together, these results indicate that PON1 might be a potential biomarker for HCC.

CRP, a protein produced by the liver, is widely used as a marker of systemic inflammation. Recent studies have indicated that it might be associated with the incidence and prognosis for a number of different cancers [19]. It appears that high levels of CRP might be related to the increased risk of liver cancer incidence [20]. In the current study, however, we found that CRP levels were decreased in the serum of HCC patients as measured by iTRAQ. This result seems to be consistent with CRP gene expression levels in HCC tissues in TCGA dataset. But the results from ELISA could not confirm these findings, suggesting that many factors may influence serum levels of CRP. Thus, CRP may not be used as a specific marker for HCC.

In summary, we identified PON1 as a potential biomarker for HCC using iTRAQ-based serum proteomic analysis. This finding was confirmed by ELISA and supported by TCGA data. Thus, PON1 might be an important biomarker for the diagnosis and pathogenesis of HCC.

## Figures and Tables

**Figure 1:** (a) Differentially expressed serum proteins in HCC patients detected by iTRAQ. (b) Cellular components of the differentially expressed proteins. (c) Biological processes involved by the differentially expressed proteins. (d) Molecular functions of the differentially expressed proteins. (e) KEGG pathway analysis of the differentially expressed proteins.

**Figure 2:** Validation of differentially expressed proteins in HCC serum by ELISA. Serum levels of (a) alpha-1-antitrypsin (A1AT), (b) peroxiredoxin 2 (PRDX2), (c) paraoxonase 1 (PON1), and (d) C-reactive protein (CRP) in HCC patients and normal controls. ^∗∗^*P* < 0.01 vs. control.

**Figure 3:** Hepatocellular carcinoma (HCC) data of (a) alpha-1-antitrypsin (A1AT), (b) peroxiredoxin 2 (PRDX2), (c) paraoxonase 1 (PON1), and (d) C-reactive protein (CRP) expression in The Cancer Genome Atlas (TCGA) database. Data are presented as medians (interquartile range (IQR)) and compared by the Mann-Whitney rank-sum test.

**Figure 4:** The relationship between the survival of HCC patients and the expression levels of (a) alpha-1-antitrypsin (A1AT), (b) peroxiredoxin 2 (PRDX2), (c) paraoxonase 1 (PON1), and (d) C-reactive protein (CRP) in TCGA database. The expression levels were divided into the high-expression and low-expression groups based on the maximally separated Kaplan-Meier plots.

**Table 1:** Patient demographic and clinical characteristics for iTRAQ and ELISA.

Characteristics	For iTRAQ		For ELISA	
	Healthy controls (*n* = 10)	HCC (*n* = 10)	Healthy controls (*n* = 20)	HCC (*n* = 20)
Gender				
Male	9	9	15	12
Female	1	1	5	8
Age (years, mean ± SD)	56.3 ± 15.0	52.5 ± 10.0	52.5 ± 12.0	59.5 ± 11.8
Coexistences (*n*)				
Hypertension	2	1	4	2
Diabetes	2	2	5	6
Smoking	2	3	4	6
Drinking	3	3	5	7
AFP (ng/ml, medians, IQR)	NA	246.2 (7.4, 356.3)	NA	15.54 (4.7, 255.3)
Child-Pugh				
A	NA	4	NA	11
B	NA	6	NA	9
Tumor size (mm, mean ± SD)	NA	58.0 ± 31.9	NA	51.3 ± 34.5
Differentiation degree				
I–II	NA	4	NA	6
II–III	NA	5	NA	10
III–IV	NA	1	NA	4

**Table 2:** List of the 41 differentially expressed proteins in HCC.

No.	Accession	Description	Coverage	Proteins	Unique peptides	Fold change cancer/normal
1	B2R950	cDNA, FLJ94213, highly similar to Homo sapiens pregnancy zone protein (PZP), mRNA	9.99	6	9	0.5155859
2	P01023	Alpha-2-macroglobulin	41.93	7	42	1.9621536
3	A8K5T0	cDNA FLJ75416, highly similar to Homo sapiens complement factor H (CFH), mRNA	51.34	5	1	1.2850993
4	P02656	Apolipoprotein C-III	34.34	2	3	0.661148
5	P01009	Alpha-1-antitrypsin	26.56	18	10	1.7751413
6	B0AZL7	cDNA, FLJ79457, highly similar to insulin-like growth factor binding protein complex acid labile chain	35.87	3	18	0.7544295
7	A8K2T4	cDNA FLJ78207, highly similar to human complement protein component C7 mRNA	50.77	6	2	1.6921352
8	P06727	Apolipoprotein A-IV	72.22	38	25	1.3346624
9	Q6LAN8	Collagen type I alpha 1 (fragment)	1.68	3	2	0.3289969
10	P27169	Serum paraoxonase/arylesterase 1	18.87	10	6	0.7979568
11	Q86TT2	Full-length cDNA clone CS0DI019YF20 of the placenta of Homo sapiens (human) (fragment)	24.58	20	5	1.3549255
12	A6XND1	Insulin-like growth factor binding protein 3 isoform b	13.31	18	3	0.8091975
13	K7ER74	Apolipoprotein C-IV	33.15	6	5	0.7221412
14	H3BRJ9	Cholesteryl ester transfer protein	3.5	5	1	0.7701269
15	P0CG05	Ig lambda-2 chain C regions	50.94	47	3	1.2929291
16	K7ERI9	Truncated apolipoprotein C-I (fragment)	23.38	6	2	0.6776806
17	B2R773	cDNA, FLJ93312, highly similar to Homo sapiens adipose most abundant gene transcript 1 (APM1), mRNA	6.15	2	1	1.2836387
18	Q8N567	Zinc finger CCHC domain-containing protein 9	12.92	1	1	2.205296
19	P51884	Lumican	40.24	2	12	1.2781468
20	D3JV41	Thrombocidin-2 antimicrobial variant (fragment)	38.1	4	5	0.7778097
21	Q59GZ2	PLEK protein variant (fragment)	1.95	2	1	0.7092328
22	Q5T0R7	Adenylyl cyclase-associated protein (fragment)	7.47	14	1	0.8056854
23	P02741	C-reactive protein	23.66	3	6	0.7119999
24	Q68CK4	Leucine-rich alpha-2-glycoprotein	43.8	2	1	0.7878539
25	P02747	Complement C1q subcomponent subunit C	15.92	1	3	1.2504316
26	B4DTB1	cDNA FLJ52936, weakly similar to tropomyosin alpha-4 chain	20.78	35	2	0.7363925
27	Q7LC44	Activity-regulated cytoskeleton-associated protein	2.78	1	1	1.4207039
28	D6R904	Tropomyosin alpha-3 chain	23.16	37	1	0.8191275
29	I2D5I8	Apolipoprotein M (fragment)	15.12	4	2	0.7276038
30	Q6NSB4	HP protein	9.61	8	3	0.8037301
31	J3KRP0	Beta-Ala-His dipeptidase	7.76	4	3	0.8289956
32	B7Z590	Cadherin-13	3.41	3	1	1.295513
33	A6NIW5	Peroxiredoxin 2, isoform CRA_a	19.85	3	2	1.2729786
34	C9JUM4	EGF-containing fibulin-like extracellular matrix protein 1 (fragment)	20.97	8	1	1.3872657
35	P08603	Complement factor H	52.15	7	2	0.7693435
36	K7EJ44	Profilin 1, isoform CRA_b	26.92	2	2	0.7312391
37	B2RA39	cDNA, FLJ94686, highly similar to Homo sapiens complement factor H-related 5 (CFHL5), mRNA	3.87	4	1	0.803087
38	P01011	Alpha-1-antichymotrypsin	40.19	4	14	0.802004
39	B2RAL6	cDNA, FLJ94991, highly similar to Homo sapiens integrin, alpha L (antigen CD11A (p180), lymphocyte function-associated antigen 1, alpha polypeptide) (ITGAL), mRNA	0.6	2	1	0.8038053
40	J3QSE5	Phosphatidylcholine-sterol acyltransferase (fragment)	9.8	4	2	0.7909272
41	B4E1C4	cDNA FLJ51179, highly similar to vitamin K-dependent protein C (EC 3.4.21.69)	16.63	16	4	0.8316701

## Data Availability

The data used to support the findings of this study are available from the corresponding author upon request (Dr. Han S.: shan87@xjtu.edu.cn).
